The article "Relative Ectopic Kidney Function Quantification Using DMSA Tomoscintigraphy Modality" was published in 2020. Journal: J Healthc Eng.

# Relative Ectopic Kidney Function Quantification Using DMSA Tomoscintigraphy Modality

**DOI:** 10.1155/2020/6092305

**Published:** 2020-05-26

**Authors:** Ines Njeh, Kalil Chtourou, Ahmed BenHamida

**Affiliations:** ^1^Advanced Technologies for Medicine and Signals (ATMS), Sfax, Tunisia; ^2^Higher Institute of Computer Science and Multimedia of Gabes, Gabes University, Gabes, Tunisia; ^3^Department of Nuclear Medicine, Habib Bourguiba University Hospital, Sfax, Tunisia; ^4^National Engineering School of Sfax, Sfax University, Sfax, Tunisia

## Abstract

The ectopic renal function estimation based on a manual region of interest (ROI) extraction could be considered as time consuming. It could also affect the clinical interpretation and thus deviate the therapeutic attitude. For this purpose, we propose an advanced tool to evaluate such function through the dimercaptosuccinic acid (DMSA) kidney scintigraphy scans. *Methods*. The proposed study has been performed on one hundred patients (fifty cases with normal kidneys and fifty cases with ectopic kidneys). We present our segmentation problems as several cost functions' optimization, each containing two terms: (i) a distribution matching prior, which evaluates a global similarity between distributions, and (ii) a smoothness prior to avoid the occurrence of small, isolated regions in the solution. Obtained following recent bound-relaxation results, the optima of the cost functions yield each kidney region in near real time. The Dice Metric (DM), the Jaccard Index (JI), and the correlation parameter have been adopted as validation parameters in order to evaluate the segmentation results. The obtained relative function of both kidneys has been then compared with that evaluated in clinical routine (planar projection) and then validated statistically by the Bland–Altman plots and the Interclass Correlation Coefficient (ICC). *Results*. Compared to the expert's manual kidney segmentation, the obtained results have been judged to be acceptable for clinical use with high Mean Dice Metric (MDM) value and high Jaccard Index (JI). The evaluated relative renal function has been different from those calculated by the projection planar method usually used in clinical routines. *Conclusion*. The proposed system could efficiently extract the renal region. The relative function estimation could be considered as more accurate. In fact, the background noise correction and the attenuation phenomenon, which could yield an error measure for renal ectopia, have been avoided. Our clinical staff members have validated the results and have suggested using such tool in their clinical routines.

## 1. Introduction

Kidney scintigraphy, also called “renal scan,” is usually used to explore the relative renal function. It could be adopted especially to evaluate kidneys' anatomy and to decide whether they are running correctly. Such modality uses a special camera, a computer, and different radiopharmaceuticals which could be defined as small amounts of radioactive materials [1]. However, this medical imaging technique could be performed with several radiopharmaceuticals such as technetium-99m dimercaptosuccinic acid (99mTc-DMSA), technetium-99m diethylenetriaminepentaacetic acid (99mTc-DTPA), technetium-99m mercaptoacetyltriglycine (99mTc-MAG3), iodine 131 orthoiodohippurate (OIH), and more recently technetium-99m ethylenedicysteine (99mTc-EC) [2]. In fact, the use of the DMSA as a static renal agent could be considered as the highest predictable method in order to evaluate the relative renal function [3]. Such exploration could be corrupted in the case of an ectopic kidney. Indeed, renal ectopia could be defined as an inborn abnormality where a kidney could be located above, below, or even on the opposite side of its conventional location. An ectopic kidney could be considered as a birth defect in which a kidney is located in an abnormal position. In fact, a fetus's kidneys first develop as small buds in the lower abdomen inside the pelvis. During the first 8 weeks of growth, the fetus's kidneys slowly move from the pelvis to their normal position in the back near the rib cage. When the kidney stays in the pelvis, it is called a pelvic kidney. If the kidney crosses to the other side of the body, it is called crossed renal ectopia. People with an ectopic kidney have no complaints. In other cases, the ectopic kidney may create urinary problems, such as urine blockage, infection, or urinary stones. One in ninety people could be affected by this anomaly [4]. The renal scintigraphy could be perturbed by several incidents such as the patient movement, the Compton diffusion, and the attenuation which could be considered as the most important disturbing factor. Unfortunately, the spine and the iliac bone could significantly attenuate the emitted photon in the case of an ectopic kidney. As a consequence, the geometric mean method usually used to correct such attenuation could be considered as insufficient. On the other hand, the activity recorded in the renal area could be assimilated to the sum of two activities: the first one is related to the tracer amount present in the kidney, and the other is due to the background noise of the kidneys' surrounding structure. As a consequence, the relative function's evaluation could be corrupted. In order to avoid these limitations, we propose a new algorithm to evaluate the relative renal function based on the kidney scan quantification. In fact, a segmentation algorithm has been used in order to delimitate each region of interest (ROI) followed by a renal count process. Based on the obtained results, we could then compute the relative function. Several researchers have investigated the use of scintigraphy scans to delimit the renal region. The authors in [5] have proposed a 3D appearance-guided deformable boundary to extract the kidneys' region. A fully automatic approach for kidney region extraction based on a multiagent system has been improved by Aribi et al. [6]. This algorithm incorporates supervisor and exploratory agents provided by the spatiotemporal points and utilizes a fast marching method in order to communicate among agents. Thresholding techniques have been adopted by several researchers. The single-threshold method has been adopted by [7], but it has been applied only in high contrast. Double threshold approach has been developed by [8] in order to identify kidney region based on a manually identified center. Landgren et al. [9] have proposed an automatic thresholding algorithm dedicated to kidney segmentation through a scintigraphy scan. However, the thresholding-based approaches have several limitations when detecting the kidney region on low contrast images especially in the case of low renal function patients. A semiautomatic ROI detection method has been presented by [10]. In fact, the manually rectangular ROI and the corresponding background area between the kidneys have been placed for each kidney. Tian et al. [11] have proposed a semiautomatic renal region of interest approach in order to evaluate the GRF estimation. In order to achieve accurate ROI detection and to avoid human intervention, fully automatic approaches have been developed. The authors in [12] present a fully automated kidney extraction based on a shape prior constrained level set algorithm in order to achieve an accurate Glomerular Filtration Rate (GFR) estimation through nuclear medicine imaging using 99mTc diethylenetriaminepentaacetic acid (99mTc-DTPA). The segmentation process has been preceded by a preprocessing step. The authors in [13] have developed a fully automatic renal ROI estimation system based on the temporal changes in intensity counts, intensity-pair distribution image contrast enhancement method, adaptive thresholding, and morphological operations that can locate the kidney area and obtain the GFR value from a (99m)Tc-DTPA renogram. The study in [14] presents the AUTOROI algorithm which has been developed to totally automatically detect whole-kidney contours and generate renal ROI for the extraction of the quantitative measurements used in the interpretation of Tc-mercaptoacetyltriglycine (Tc-MAG3) renograms.

The aim of this study is to present a more accurate relative ectopic renal function evaluation tool compared to those obtained in clinical routines. The fully automatic ROI extraction offers the possibility of better quantifying the kidney region by avoiding the background noise corruption and the attenuation phenomenon.

The main contributions of this research are as follows:

  It is the first work dealing with the ectopic kidney anomalies through the dimercaptosuccinic acid (DMSA) kidney scintigraphy scans
  The proposed algorithm is fully automatic and presents great performance
  The use of such algorithm could modify the action to be conducted

## 2. Materials and Methods

### 2.1. Subjects

Fifty normal cases (24 men and 26 women; age range 29–60) and fifty ectopic patients (29 men, 21 women; age range, 31–55) who have been subjected to kidney scintigraphy with 99mTc-DMSA in order to diagnose their kidney disorders have been considered in this study. Fifty patients had a normal scan, and the other fifty exhibited an ectopic kidney.

### 2.2. Imaging Procedures

A good hydration has been suggested before and after radiotracer injection. Thirty-five minutes after the oral consumption of water or intravenous solution administration, the patient has been injected with radioactive technetium-99m combined with dimercaptosuccinic acid (DMSA). After 2–6 hours, the static imaging could be performed using a gamma camera. Imaging could take nearly 5–10 minutes. The tomographic acquisition has been considered, in this work, since it allows us to obtain a projection in three plans. Such acquiring could give us a more precise analysis of the radiopharmaceuticals repartition on each kidney.

### 2.3. Standard Method

In clinical routines, the planar quantification technique has been adopted to compute the relative renal function through the anterior and the posterior projection. However, the registered renal computation could be considered as different from the real activity fixed on the renal cortex. In fact, the background as well as the attenuation phenomenon due to the structure situated between the kidney and the gamma camera detector could be responsible for this difference. For this reason, we should realize some correction in order to correct the relative renal function value.

#### 2.3.1. Background Noise Correction

The extrarenal and the intrarenal component could be considered as the two principal renal background components. The extrarenal component, known also as interstitial, could include extravascular as well as intravascular parts. The intravascular part could drop quickly during the first minutes after the injection [15]. At the same time, the extrarenal background could moderately grow [16]. The two components could decrease or flatten depending on the extrarenal region vascular structure [17].

As illustrated in Figure 1, manually created regions of interest (ROI) have been drawn on both posterior and anterior projections wrapping each renal ROI and its corresponding background noise [18]. *Q*_b_ represents the total count of each kidney, and *Q*_F_ represents the background noise count.

The corrected total renal count could be computed by

(1) $$\begin{array}{c} Q_{\text{BC}}=Q_{\text{b}}-N_{Q_{\text{b}}}*\frac{Q_{\text{F}}}{N_{Q_{\text{F}}}}, \end{array}$$

where *Q*_BC_ represents the corrected total renal count, *Q*_b_ represents the total renal count, *N*_*Q*_b__ represents the pixel number of the renal region of interest, *N*_*Q*_F__ represents the pixel number of the background region, and *Q*_F_ represents the background region count.

#### 2.3.2. Attenuation Correction

Right and left kidneys are not localized in the same depth. Generally, the left kidney is closer to the posterior side compared to the right kidney. Such difference in depth could yield corrupted relative renal function quantification [19]. In clinical routines, the mean geometric method has been used in order to correct the kidney depth based on the anterior and the posterior projection [20]. The ameliorated renal count after the attenuation correction could be computed by

(2) $$\begin{array}{c} Q_{\text{AC}}=\sqrt{C_{\text{ant}}*C_{\text{post}}}*e^{\mu \text{d}}, \end{array}$$

where  *Q*_AC_ represents the attenuation corrected renal count, *C*_ant_ represents the anterior saved count, *C*_post_ represents the posterior saved count, *μ* is the attenuation coefficient of the soft part and is fixed to 1.43 cm^−1^, and *d* is the patient's kidney depth.

The renal depth (*d*) has been calculated from the difference between the kidney region gravity center and the two mean points' position in both anterior and posterior direction [21].

#### 2.3.3. Relative Renal Function Quantification

After the attenuation correction (AC), the relative renal function quantification could be computed as follows:

(3) $$\begin{array}{c} {\text{RF}}_{\text{right}}=\frac{Q_{\text{AC}}^{\text{right}}}{Q_{\text{AC}}^{\text{right}}+Q_{\text{AC}}^{\text{left}}}*100,\\ {\text{RF}}_{\text{left}}=\frac{Q_{\text{AC}}^{\text{left}}}{Q_{\text{AC}}^{\text{right}}+Q_{\text{AC}}^{\text{left}}}*100, \end{array}$$

where *a*_AC_^right^  and *Q*_AC_^left^ are, respectively, the right renal count and the left renal count obtained after the attenuation correction (AC).

### 2.4. Planar Projection Limitation

The geometric mean method could be considered as inconvenient for the planar projection. In fact, such method assumes that the traversed structures are always homogeneous and identical for the two kidneys. Such supposition could be considered as inappropriate especially in the ectopic kidneys case. Indeed, the bone structures (iliac bone and lumbar spine) are more attenuating than the soft parts [22]. In addition, this technique estimates that the posterior depth traversed by the emitted photons is always identical (abdominal depth) for both kidneys. Such condition could not be satisfied in the case of pelvic ectopic kidney. That is why we could conclude that the mean geometric technique is unreliable in the case of ectopic kidney. For this reason, we have adopted a new technique in order to evaluate the relative renal function based on the renal region extraction through tomoscintigraphy scans. In fact, such procedure could eliminate the planar projection limitation and thus provide a more accurate diagnosis.

### 2.5. ROI Extraction

The proposed segmentation approach has been used previously to segment brain tumor on both 2D [23] and 3D [24] Magnetic Resonance Imaging. In this work, we have adopted the algorithm in order to extract the kidney region from the scintigraphy scans.

The proposed algorithm does not require an excessive training. It utilizes only the image information. We define Φ_s_ as a fragment of the total image domain including the kidney region.  Figure 2 illustrates a typical example in which Φ_s_ represents the zone containing the kidney and $\bar{\Phi_{\text{s}}}$ the tissues surrounding the kidney whose intensity distribution most closely matches the defined model *D*. The obtained zone represents the complement of the kidney region in Φ_s_, thus the kidney region which is our objective. We describe the problem as energy function optimization containing (1) an intensity distribution matching term which computes a global similarity among nonparametric distributions and (2) a smoothness term used to inhibit the development of limited isolated zone in the result. The algorithm requires very little iteration to converge, thus offering a nearly real-time simulation.

In order to define $\bar{\Phi_{\text{s}}}$ and Φ_s_, we should divide the image into two parts. The user should only choose between three options: “right kidney,” “left kidney,” and “two kidneys.” For the first and the second options, a vertical line has been used in order to define the region containing the kidney and the region including only the safety parts by dividing the image into two different parts. For the last option, a horizontal line has been chosen. The division process has been achieved automatically based on the user choice as illustrated in Figure 3.

Figure 4 illustrates the flowchart of the proposed algorithm adopted to extract the kidney region through the DMSA tomoscintigraphy modality.

### 2.6. Formulation

We consider *I*_*i*_=*I*(*i*) :  Φ_s_  ⊂ *ℝ*^2^  as an image function representing a fixed domain  Φ_s_.  Φ_s_ represents a part from the image which contains the kidney region (corresponding to the left hand part in Figure 2). Let *M* be the total image domain. We could define $\;\bar{\Phi_{\text{s}}}=M/\Phi_{\text{s}}$ designating the complement region of  Φ_s_ in *M*. D represents the distribution kernel density estimation of an image data inside $\bar{\Phi_{\text{s}}}$ expressed as follows:

(4) $$\begin{array}{c} \forall \;x\in \;\mathbb{R},D\left(x\right)=\frac{\sum_{i\in \bar{\Phi_{\text{s}}}}K_{x}\left(I_{i}\right)}{A\left(\bar{\Phi_{\text{s}}}\right)}, \end{array}$$

where $A\left(\bar{\Phi_{\text{s}}}\right)$ represents the pixel number in the region $\bar{\Phi_{\text{s}}}\subset M$ and *K*_*x*_(·) is the usually Gaussian kernel function:

(5) $$\begin{array}{c} K_{x}\left(y\right)=\frac{1}{\sqrt{2\pi \sigma^{2}}}\exp\left(-\frac{x-y}{2\sigma^{2}}\right). \end{array}$$

We could consider *K*_*x*_(·) as a Dirac function in order to obtain a normalized histogram. *D* represents the prior model that includes the totality of statistical information about the part which does not contain the kidney. The principal step of the algorithm resides in detecting within Φ_s _ (i.e., the part which does not contain the kidney) a region *E* whose intensity distribution most closely matches the model D (right hand side in Figure 2). Such region provides the safety tissues in Φ_s _ and, as a consequence, the kidney region which is our target.

The problem could be stated as the minimization of a discrete function conducive to binary labeling *L*_*x*_=*L*_*x*_ : Φ_s _⟶{0,1}, characterizing a variable partition of Φ_s _ : *E*={*x* ∈ *X* /*L*_*x*_=1} matching the safety tissues and its counterpart in Φ_s _, $\bar{E}=\left\{x\in X\;/L_{x}=0\;\right\}=\Phi_{\text{s }}\backslash E$ corresponding to the kidney region.

To obtain the optimal labeling, we should minimize a global cost function including a distribution matching constraint based on the Bhattacharyya measure and a smoothness constraint. In order to introduce the cost function, we should suggest the succeeding notations for any binary labeling *L*_*x*_=*L*_*x*_ :  Φ_s_⟶{0,1}:

- *E* is the variable region provided by *E*={*x* ∈ *X*/*L*_*x*_=1 }  ⊂ Φ_s_ .
- *P*_*E* _ could be defined as the Kernel Density Estimate (KDE) of the image data distribution inside the region *E*={*x* ∈ *X*/ *L*_*x*_=1 }

(6) $$\begin{array}{c} P_{E}\left(x\right)=\frac{\sum_{x\in E}K_{x}\left(I_{x}\right)}{A\left(E\right)},\;\forall \;x\in X. \end{array}$$

(iii) *B*(*f*, *g*) is the Bhattacharyya coefficient used to evaluate the overlap amount between two different distributions *f* and *g*:

(7) $$\begin{array}{c} B\left(f,g\right)=\sum_{x\in X}\sqrt{f\left(z\right).g\left(z\right)}. \end{array}$$

The algorithm resides in detecting the optimal labeling *L*^opt^ which minimizes the presented cost function:

(8) $$\begin{array}{c} L^{\text{opt}}=\underset{L}{\min}C\left(L\right), \end{array}$$

with

(9) $$\begin{array}{c} C\left(L\right)=S\left(P_{E}\;,\;D\right)+\gamma \;E\left(L\right)\\ \text{ s.t }E=\left\{\frac{x\in P}{\;L_{x}=1}\right\}. \end{array}$$

*S* could be defined as the distribution matching constraint obtained by the negative Bhattacharyya coefficient:

(10) $$\begin{array}{c} S\left(P_{E},D\right)=-B\left(P_{E},D\right)=-\sum_{x\in X}P_{E}\left(x\right)\cdot D\left(x\right). \end{array}$$

*E*(*L*) is a regularization prior used in order to minimize the boundary partition length [25].

(11) $$\begin{array}{c} E\left(L\right)=\sum_{\left\{x,y\right\}\in N}S_{x,y}\;\delta_{L_{x}=L_{y}}, \end{array}$$

with

(12) $$\begin{array}{c} \delta_{i\neq j}=\left\{\begin{array}{cc} 1, & \text{if }i\neq j,\\ 0, & \text{if }i=j, \end{array}\right.\\ S_{i,j}=\frac{1}{\left\|i-j\right\|}. \end{array}$$

*N* could be defined as some neighborhood system including all pairs {*i*, *j*} of neighboring elements in Φ_s_. The regularization prior prevents the small isolated regions development in the solution.  *γ* represents a positive constant that adjusts the relative distribution matching contribution and the regularization term.  *L*^opt^ yields then an optimal boundary-smooth region, *E*^opt^={*x* ∈ *X*/*L*_*x*_^opt^=1}, whose intensity distribution most closely matches D. The obtained optimal region corresponds to the tissues region in Φ_s_. As a consequence, the kidney region could be finally deduced from  *L*^opt^ as follows:

(13) $$\begin{array}{c} E^{\text{Kidney}}=\Phi_{\text{s}}\backslash E^{\text{opt}}=\left\{\frac{x\varepsilon X}{L_{x}^{\text{opt}}=0}\;\right\}. \end{array}$$

## 3. Results

### 3.1. Quantitative Evaluation

One senior clinician who has several years of experience in renal evaluation manually drew the region of interest (ROI) as in the routine clinical procedure. Such manual segmentation has been considered as a ground truth. In order to validate the obtained results, quantitative evaluation and statistical analysis have been conducted in order to assess the performance of the proposed tool. In fact, The Dice Metric (DM) parameters as well as the Jaccard Index (JI) have been used to compare the obtained segmentation result with the manual ROI extraction provided by the expert.

### 3.2. Dice Metric

For the segmentation results' evaluations, the Dice Metric (DM) has been adopted as a validation parameter. DM is frequently used, in the literature, to gauge the closeness between the automatic segmentation results and the reference (ground truth or expert manual segmentation) [26, 27]. DM could be defined as follows:

(14) $$\begin{array}{c} \text{DM}=\frac{V_{\text{AM}}}{V_{\text{A}}+V_{\text{M}}}, \end{array}$$

where *V*_A_, *V*_M_, and *V*_AM_ represent, respectively, the automatically segmented region, the expert manual segmentation, and the intersection between them. DM has a value in [0, 1]. 1 indicates a perfect similarity between the two segmentations. A higher DM validates the algorithm performance.

### 3.3. Jaccard Index Coefficient

A second validation parameter has been adopted in this work in order to assess the proposed segmentation algorithm performance. The Jaccard Index (JI) [28] has been usually used in order to measure the similarity and the overlap between the obtained results and the manual segmentation. It could be defined as

(15) $$\begin{array}{c} \text{JI}=\frac{\left|\;V_{\text{A}}\cap V_{\text{M}}\right|}{\;\left|V_{\text{A}}\cup V_{\text{M}}\right|}, \end{array}$$

where *V*_A_ and  *V*_M _ represent the automatically segmented region and the expert manual segmentation. The Jaccard Index (JI) could have a value in [0, 1]. 1 indicates a perfect match between the two segmentations. A higher Jaccard Index (JI) affirms the algorithm performance.

### 3.4. Statistical Analysis

The correlation [29] between the manual segmentation and the obtained result has been evaluated in order to verify the performance of the proposed method. The Bland–Altman [30] plots have been drawn and the Interclass Correlation Coefficient (ICC) has been computed in order to compare the obtained relative ectopic kidney function with those computed by the planar quantification usually adopted in clinical routines.

The MedCalc software has been used to realize the statistical analysis during this research.

### 3.5. Ectopic Kidney Segmentation

In this section, we report the segmentation results obtained by the application of the proposed methodology to the clinical dataset. Several visual typical illustrations through different ectopic kidney scans will be also presented. The Mean Dice Metric (MDM), the Mean Jaccard Index (MJI), and the correlation have been adopted as validation parameters in order to evaluate the proposed algorithm performance.

Figure 5 shows the obtained result of an ectopic kidney patient. The blue curve represents the obtained right kidney boundary, the red line corresponds to the left kidney boundary, and the yellow curve involves the manual segmentation performed by an expert. The obtained binary mask for the considered ROI is represented by Figure 5(c). The ROI extraction illustrated by Figure 5(d) will be used to evaluate the relative ectopic kidney function. The proposed algorithm requires only four iterations and grants automatic segmentation in 0.35 s.

Figure 6 illustrates an ectopic and hydronephrosis patient. The blue curve represents the obtained right kidney boundary, the red line corresponds to the left kidney boundary, and the yellow curve involves the manual segmentation performed by an expert. The obtained binary mask for the considered ROI is represented by Figures 6(c) and 6(g). The ROI extraction illustrated by Figures 6(d) and 6(h) will be used to evaluate the relative ectopic kidney function. The proposed algorithm requires only three iterations and grants automatic segmentation in 0.25 s.

We could conclude that the proposed algorithm requires few iterations (less than 5) to handle a kidney scan in near real time (less than 0.5 seconds).

Table 1 illustrates the Mean Dice Metric (MDM) and the Mean Jaccard Index (MJI) through the different right kidney of clinical cases (fifty normal patients and fifty ectopic patients).

We have computed the Dice Metric (DM) parameter as well as the Jaccard Index (JI) between the obtained result and the manual segmentation for each patient on all slices, and we have, then, evaluated the mean value on the patient's totality (50 normal patients and 50 ectopic cases). We could notice that the proposed method presents a great performance since the MDM is about 0.9874 for normal patients and 0.9725 for ectopic cases. The MJI is 0.9741 for normal patients and 0.9654 for ectopic patients, which could validate the performance of the proposed algorithm.

Table 2 illustrates the Mean Dice Metric (MDM) and the Mean Jaccard Index (MJI) through the different left kidney of clinical cases (fifty normal patients and fifty ectopic patients).

We have computed the Dice Metric (DM) parameter as well as the Jaccard Index (JI) for the obtained result and the manual segmentation for each patient on all slices, and we have, then, evaluated the mean value on the patient's totality (50 normal patients and 50 ectopic cases). We could notice that the proposed method presents a great performance since the MDM is about 0.9877 for normal patients and 0.9791 for ectopic cases. The MJI is 0.9798 for normal patients and 0.9685 for ectopic patients, which could validate the performance of the proposed algorithm.

In order to assess the performance of the proposed segmentation algorithm, we have computed the correlation between the obtained result and the manual segmentation. We have chosen the central slice and we have computed the intensity in the ROI part.

The scatter plot of the ROI intensity obtained using both the manual segmentation and the automated method for the right kidney of the normal patients is shown in Figure 7. The correlation between these two approaches was found to be *y* = 0.975 − 0.00755 (*r* = 0.97).

The scatter plot of the ROI intensity obtained using both the manual segmentation and the automated method for the left kidney of the normal patients is shown in Figure 8. The correlation between these two approaches was found to be *y* = 1.007*x* − 1.037 (*r* = 1).

The scatter plot of the ROI intensity obtained using both the manual segmentation and the automated method for the right kidney of the ectopic patients is shown in Figure 9. The correlation between these two approaches was found to be *y* = 1.000*x* − 0.981 (*r* = 1).

The scatter plot of the ROI intensity obtained using both the manual segmentation and the automated method for the left kidney of the ectopic patients is shown in Figure 10. The correlation between these two approaches was found to be *y* = 0.997*x* − 0.173 (*r* = 1).

### 3.6. Relative Function Evaluation

As mentioned in the previous section, the relative function evaluation could affect the clinical prognosis especially in ectopic kidney. In this part, we present the obtained value by applying the proposed methodology and the results provided by the planar quantification method.

A statistical analysis has been performed, using the MedCalc software, in order to assess the performance of the proposed method especially in the case of ectopic kidney. In fact, the Bland–Altman plots comparing the obtained result and those computed by the planar quantification have been drawn. The Interclass Correlation Coefficient (ICC) [31] has been also computed in order to compare the obtained relative function and those computed by the planar quantification.

Figure 11 illustrates the Bland–Altman plot for the right kidney in fifty normal cases. We could notice that the obtained relative function and those obtained by the planar quantification method could be considered as similar.

Table 3 illustrates the Interclass Correlation Coefficient (ICC) of the obtained relative function and the planar quantification method for the right kidney in fifty normal cases. The ICC value is nearly 1, which could verify the similarity between the considered values.

Figure 12 illustrates the Bland–Altman plot for the left kidney in fifty normal cases. We could notice that the obtained relative function and those obtained by the planar quantification method could be considered as similar.

Table 4 illustrates the Interclass Correlation Coefficient (ICC) of the obtained relative function and the planar quantification method for the left kidney in fifty normal cases. The ICC value is nearly 1, which could verify the similarity between the considered values.

Figure 13 illustrates the Bland–Altman plot for the right kidney in fifty ectopic cases. We could notice that the obtained relative function and those obtained by the planar quantification method could be considered as different, which could modify the action to be conducted in clinical routines.

Table 5 illustrates the Interclass Correlation Coefficient (ICC) of the obtained relative function and the planar quantification method for the right kidney in fifty ectopic cases. The ICC value is not near 1, which could confirm the difference between the obtained results and the values obtained by the planar quantification method.

Figure 14 illustrates the Bland–Altman plot for the right kidney in fifty ectopic cases. We could notice that the obtained relative function and those obtained by the planar quantification method could be considered as different, which could modify the action to be conducted in clinical routines.

Table 6 illustrates the Interclass Correlation Coefficient (ICC) of the obtained relative function and the planar quantification method for the left kidney in fifty ectopic cases. The ICC value is not near 1, which could confirm the difference between the obtained results and the values obtained by the planar quantification method.

We could notice the difference between the obtained values and the planar quantification results. Such difference could explain the advantage of the proposed method. In fact, it provides a more accurate evaluation since it is not affected by the background noise and the attenuation phenomenon.

## 4. Discussion

In this work, we have adopted corrected tomoscintigraphic renal scans. In fact, a specific attenuation coefficient card for each patient has been obtained during the acquisition process. In clinical routines, the planar quantification has been used to compute the relative kidney function of both normal and ectopic kidney. It uses the anterior and the posterior projection which are corrected by the mean geometric method. An attenuation phenomenon consideration as well as a background correction has been suggested in order to reduce the error value. The relative renal function computed by the planar quantification technique has been provided by our clinical staff in order to make a comparative study. However, the mean geometric method supposes that the traversed anteroposterior thickness (abdominal thickness) could be considered as similar for the two kidneys. It considers that the attenuation coefficient is constant, and it is *μ*=1.45 cm^−1^. This condition is only available for the normal patients when the kidneys are located in their original places. As a consequence, the computation of the relative renal function by the planar quantification could be considered as acceptable (Tables 3 and 4). However, this method will not be performed in the case of ectopic kidney since the structure thickness traversed by the anterior and the posterior photons is inhomogeneous and did not present the same thickness for the two kidneys (Tables 5 and 6). The patient presented as Case 3 had an ectopic and hydronephrosis right kidney. The scatter and the background noise values have been significantly increased by the radioactive urine stasis. The difference between the value obtained by the proposed method and that by the planar quantification method is nearly 7%. Such difference could change the therapeutic attitude. We could conclude that the proposed method based on scintigraphy scan segmentation could present more advantages than the planar quantification usually used in clinical routines, since it helps to avoid the attenuation phenomenon and reduce the background noise. As a consequence, we recommend the use of the proposed technique in clinical routines especially in the case of ectopic and even hydronephrosis kidneys.

## 5. Conclusion

In this work, we have proposed an advanced approach to evaluate the relative renal function through the 99mTc-DMSA tomoscintigraphic scans in near real time. The segmentation results have been validated by our clinical staff. The Mean Dice Metric (MDM) parameter as well as the Mean Jaccard Index (MJI) has been adopted to compare the manual expert segmentation and the obtained result. The correlation parameter has been computed in order to statistically validate the obtained segmentation results. The higher MDM, the higher MJI, and the higher correlation values could thus verify the performance of the proposed segmentation algorithm. The proposed algorithm aims to calculate the relative renal function without the influence of the attenuation phenomenon and the background noise problem which could be considered as error source in the planar quantification technique usually used in clinical routines. The obtained results have been statistically validated by the Bland–Altman plots and by the Interclass Correlation Coefficient (ICC) computation. The use of such algorithm could change the therapeutic attitude especially in the case of ectopic and even hydronephrosis kidney.

## Figures and Tables

**Figure 1:** Background noise illustration.

**Figure 2:** Main steps of the proposed algorithm.

**Figure 3:** Illustration of the definition of $\bar{\Phi_{\text{s}}}$ and  Φ_s_ region: (a) left kidney, (b) two kidneys, and (c) right kidney.

**Figure 4:** Flowchart of the proposed kidney segmentation algorithm.

**Figure 5:** Ectopic kidney segmentation: (a) input image; (b) segmented image, where the right kidney is delimited by the blue line, the left kidney is delimited by the red line, and the manual segmentation is represented by the yellow line; (c) binary ROI extraction; (d) ROI extraction.

**Figure 6:** Ectopic and hydronephrosis kidney segmentation: (a, e) input images; (b, f) segmented images, where the right kidney is delimited by the blue line, the left kidney is delimited by the red line, and the manual segmentation is represented by the yellow line; (c, g): binary ROI extraction; (d, h) ROI extraction.

**Figure 7:** Correlation of the manual segmentation and automated segmentation methods for the right kidney of the normal patients.

**Figure 8:** Correlation of the manual segmentation and automated segmentation methods for the left kidney of the normal patients.

**Figure 9:** Correlation of the manual segmentation and automated segmentation methods for the right kidney of the ectopic patients.

**Figure 10:** Correlation of the manual segmentation and automated segmentation methods for the left kidney of the ectopic patients.

**Figure 11:** Bland–Altman plot for the right kidney in fifty normal cases.

**Figure 12:** Bland–Altman plot for the left kidney in fifty normal cases.

**Figure 13:** Bland–Altman plot for the right kidney in fifty ectopic cases.

**Figure 14:** Bland–Altman plot for the left kidney in fifty ectopic cases.

**Table 1:** Mean Dice Metric (MDM) and Mean Jaccard Index (MJI) evaluation for both normal and ectopic patients (right kidney).

	Mean Dice Metric (MDM)	Mean Jaccard Index (MJI)
Normal patients	0.9847	0.9741
Ectopic patients	0.9725	0.9654

**Table 2:** Mean Dice Metric (MDM) and Mean Jaccard Index (MJI) evaluation for both normal and ectopic patients (left kidney).

	Mean Dice Metric (MDM)	Mean Jaccard Index (MJI)
Normal patients	0.9877	0.9798
Ectopic patients	0.9791	0.9685

**Table 3:** The Interclass Correlation Coefficient evaluation of the obtained relative function and the planar quantification method for the right kidney in 50 normal cases.

	Interclass Correlation	95% confidence interval
Single measures	0.9950	0.8451 to 0.9987
Average measures	0.9975	0.9161 to 0.9994

**Table 4:** The Interclass Correlation Coefficient evaluation of the obtained relative function and the planar quantification method for the left kidney in 50 normal cases.

	Interclass Correlation	95% confidence interval
Single measures	0.9952	0.8454 to 0.9988
Average measures	0.9976	0.9163 to 0.9994

**Table 5:** The Interclass Correlation Coefficient evaluation of the obtained relative function and the planar quantification method for the right kidney in 50 ectopic cases.

	Interclass Correlation	95% confidence interval
Single measures	0.7792	−0.01099 to 0.9483
Average measures	0.8759	−0.02223 to 0.9734

**Table 6:** The Interclass Correlation Coefficient evaluation of the obtained relative function and the planar quantification method for the left kidney in 50 ectopic cases.

	Interclass Correlation	95% confidence interval
Single measures	0.7003	−0.02173 to 0.9202
Average measures	0.8238	−0.04442 to 0.9584

## Data Availability

The data used to support the findings of this study are included within the article.

## References

[1] Taylor A., Nally J. V. (1995). Clinical applications of renal scintigraphy. *American Journal of Roentgenology*.

[2] Moran J. K. (1999). Technetium-99m-EC and other potential new agents in renal nuclear medicine. *Seminars in Nuclear Medicine*.

[3] Ardela Diaz E., Miguel Martinez B., Gutierrez Duenas J. M., Diez Pascual R., Garcia Arcal D., Dominguez Vallejo F. J. (2002). Comparative study of differential renal function by DMSA and MAG-3 in congenital unilateral uropathies. *Cirugia Pediatrica*.

[4] Shapiro E., Bauer S. B., Chow J. S. (2012). Anomalies of the upper urinary tract. *Campbell-Walsh Urology*.

[5] Shehata M., Mahmoud A., Soliman S. (2018). 3D kidney segmentation from abdominal diffusion MRI using an appearance-guided deformable boundary. *PLoS One*.

[6] Aribi Y., Wali A., Chakroun M., Alimi A. M. (2013). Automatic definition of regions of interest on renal scintigraphic images. *AASRI Procedia*.

[7] Halker R. K., Chrem Y., Galt J. R. (1996). Interoperator variability in quantitating the MAG3 renal uptake based on semiautomated and manual regions of interest. *Journal of Nuclear Medicine*.

[8] Tomaru Y., Inoue T., Oriuchi N. (1998). Semi-automated renal region of interest selection method using the double-threshold technique: inter-operator variability in quantitating ^99m^TcMAG_3_ renal uptake. *European Journal of Nuclear Medicine*.

[9] Landgren M., Sjöstrand K., Ohlsson M. (2011). An automated system for the detection and diagnosis of kidney lesions in children from scintigraphy images. *Image Analysis*.

[10] Inoue Y., Yoshikawa K., Yoshioka N. (2000). Evaluation of renal function with ^99m^Tc-MAG_3_ using semi-automated regions of interest. *Journal of Nuclear Medicine*.

[11] Tian C., Zheng X., Han Y., Sun K., Chen K., Huang Q. (2013). A semi-automated region of interest detection method in the scintigraphic glomerular filtration rate determination for patients with abnormal low renal function. *Clinical Nuclear Medicine*.

[12] Zheng X., Wei W., Huang Q., Song S., Huang G. (2019). Automated region of interest detection method in scintigraphic glomerular filtration rate estimation. *IEEE Journal of Biomedical and Health Informatics*.

[13] Lin K.-J., Huang J.-Y., Chen Y.-S. (2011). Fully automatic region of interest selection in glomerular filtration rate estimation from ^99m^Tc-DTPA renogram. *Journal of Digital Imaging*.

[14] Garcia E. V., Folks R. S., Taylor A. (2010). Totally automatic definition of renal regions of interest from ^99m^Tc-MAG_3_ renograms: validation in patients with normal kidneys and in patients with suspected renal obstruction. *Nuclear Medicine Communications*.

[15] Peters A. M., Gordon I., Evans K., Todd-Pokropek A. (1987). Background in the ^99m^Tc DTPA renogram: analysis of intravascular and extravascular components. *American Journal of Physiologic Imaging*.

[16] Decostre P. L., Salmon Y. (1990). Temporal behavior of peripheral organ distribution volume in mammillary systems: application to background correction in separate glomerular filtration rate estimation. *The Journal of Nuclear Medicine*.

[17] Moonen M., Granerus G. (1992). Subtraction of extra-renal background in ^99m^Tc-DTPA renography: comparison of various regions of interest. *Clinical Physiology*.

[18] Fleming J. S. (2006). A technique for analysis of geometric mean renography. *Nuclear Medicine Communications*.

[19] Argenta J., Brambila C. R., Silva A. M. M. D. (2010). Attenuation correction for renal scintigraphy with ^99m^Tc-DMSA: analysis between Raynaud and the geometric mean methods. *Revista Brasileira de Medicina do Esporte (RBME)*.

[20] Chroustová D., Trnka J., Šínkas V., Urbanova I., Langer J., Kubinyi J. (2016). Comparison of planar DMSA scan with an evaluation based on SPECT imaging in the split renal function assessment. *Nuclear Medicine Review*.

[21] Steinmetz A. P., Zwas S. T., Macadziob S., Rotemberg G., Shrem Y. (1998). Renal depth estimates to improve the accuracy of glomerular filtration rate. *Journal of Nuclear Medicine*.

[22] Miller C., Filipow L., Jackson S. (1995). A review of activity quantification by planar imaging methods. *Journal of Nuclear Medicine Technology*.

[23] Njeh I., Ben Ayed I., Ben Hamida A. A distribution matching approach to MRI brain tumor segmentation.

[24] Njeh I., Sallemi L., Ayed I. B. (2015). 3D multimodal MRI brain glioma tumor and edema segmentation: a graph cut distribution matching approach. *Computerized Medical Imaging and Graphics*.

[25] Boykov Y., Kolmogorov V. Computing geodesics and minimal surfaces via graph cuts.

[26] Pratsawa M., Bullitt E., Ho S., Grerig G. (2004). A brain tumor segmentation framework based on outlier detection. *Medical Image Analysis*.

[27] Ho S., Bullitt E., Gerig G. Level set evolution with region competition: automatic 3-D segmentation of brain tumors.

[28] Raimundo R., Juan M. V. (1996). The probabilistic basis of Jaccard’s index of similarity. *Systematic Biology*.

[29] Schober P., Boer C., Schwarte L. A. (2018). Correlation coefficients. *Anesthesia & Analgesia*.

[30] Bland J. M., Altman D. G. (1986). Statistical methods for assessing agreement between two methods of clinical measurement. *The Lancet*.

[31] Müller R., Büttner P. (1994). A critical discussion of intraclass correlation coefficients. *Statistics in Medicine*.

